The article "Application of Artificial Intelligence in the Intervention of Sports on Adolescent Health Risk Behavior" was retracted in 2023. Reasons: signs of a paper mill; compromised peer review; unreliable results or conclusions.

# Application of Artificial Intelligence in the Intervention of Sports on Adolescent Health Risk Behavior

**DOI:** 10.1155/2022/1594108

**Published:** 2022-04-11

**Authors:** Jin Ha

**Affiliations:** North Minzu University, Yinchuan, China

## Abstract

Through school education to intervene in the behavior of adolescent health risk behaviors students and guide students to have a correct concept of quality and health, this paper uses artificial intelligence technology to mine students' body language to analyze students' behavior in quality education dance classes, so as to achieve effective intervention for AHRB students. Before the experimental study, AHRB students and normal students were mixed into groups in a ratio of not less than 1 : 18. The results of the study showed that the implementation of intervention strategies could reduce the recurrence of various risky behaviors in adolescents. When non-AHRB students and AHRB students intervene together, there will be no adverse effects on non-AHRB students.

## 1. Introduction

As a key link in inheriting the development of human civilization, youth is the hope of the country in the future, and a healthy body is the foundation. The education and health habits formed in youth will accompany him all his life and have a lot of influence on social and economic aspects [1]. In modern society, families, schools, and society have brought great pressure and challenges to teenagers. If teenagers want to develop comprehensively, they must have good physical quality and psychological quality [2]. In adolescence, if there are no reasonable prevention and control of adolescent health, there may be many adolescents with dangerous health behavior (adolescent health risk behavior (AHRB)), such as not intentional injury behavior, intentional injury behavior, drug addiction or mental addiction behavior, dangerous behavior, unhealthy diet behavior, personality disorder behavior, susceptibility to various chronic diseases and adolescent early death or disability, even forming antisocial behavior, causing social problems, and bringing negative impact [3].

With the development of social economy, teenagers rely too much on smart devices, smoking, drinking and even taking drugs due to learning pressure or family factors, which can be effectively improved under family or school intervention. However, the family or school cannot find out in time or take effective measures after the discovery. Xia conducted a random sampling survey of 10 middle schools in Harbin, established a multivariate analysis model to investigate the health status of students, discussed the prevention and control of adolescent injury, reduced the incidence rate, and explored the health education intervention strategy [4]. Pan et al. conducted a random sample of 998 teenagers in Zhenhai District to understand the characteristics and influencing factors of AHRB and to formulate targeted preventive measures [5].

The article "Application of Artificial Intelligence in the Intervention of Sports on Adolescent Health Risk Behavior" was retracted in 2023. Reasons: signs of a paper mill; compromised peer review; unreliable results or conclusions.

In recent years, as the country pays more and more attention to the physical exercise of students, various sports activities are carried out in colleges and universities to enhance the physical fitness of young people and promote their physical and mental health, which is conducive to the overall development of young people's physical and mental health [6]. Although many colleges and universities have carried out physical exercise activities, the effect of intervention on AHPB is not obvious.

## 2. Relevant Technologies of AI Sports and AHRB Recognition Intervention

Other behaviors that may affect the health of teenagers, such as intentional injury, drowning, and other dangerous behaviors that may affect the quality of life of teenagers, such as drug addiction, lead to unexpected pregnancy or early uncontrolled sexual behavior of sexually transmitted diseases, unhealthy eating behavior, or personality disorder behaviors such as loneliness, laziness, inferiority complex, and excessive dependence.

In the current educational technology system, the early recognition and early warning technology of AHRB are not perfect, but after the first discovery of AHRB behavior, the recurrence of AHRB behavior can be effectively avoided through certain educational means. For example, the study used artificial intelligence sports to carry out a comprehensive intervention on multiple young students who had AHRB behavior at least once and achieved certain positive results.

Quality sports dance refers to physical education for ordinary schools. The purpose of quality-oriented sports dance education is not sports itself, nor does it make all students become sports dancers, but a new type of youth quality education. The dance course of quality education is quite different from the art dance course and sports dance course. This sports course model does not arrange fixed dance movements but requires students to freely express body language according to music melody and beat. Li et al., through the promotion of quality education dance in Hengshui primary schools, believe that quality education dance has a great significance to the cultivation of quality-oriented education [7]. In the early stage, the course was not effectively promoted due to the lack of evaluation mechanism, but after the relevant research gradually deepened the artificial intelligence intervention technology and analysis technology of AHRB, the quality education dance class combined with the artificial intelligence sports analysis function was used to obtain the positive intervention effect on AHRB students [8, 9]. At the same time, in view of the intervention effect of relevant research on autism and depression of quality-oriented education dance, this study delves into its intervention effect on AHRB [10].

The article "Application of Artificial Intelligence in the Intervention of Sports on Adolescent Health Risk Behavior" was retracted in 2023. Reasons: signs of a paper mill; compromised peer review; unreliable results or conclusions.

## 3. Research Contents and Investigation Methods

### 3.1. Selection and Grouping of Student Samples

As a key part of the continuation of social life and the inheritance of civilization, teenagers are also the sustenance of life, health, and spirit in the future [11]. If teenagers have various dangerous behaviors and parents, schools, and society do not intervene early, they will endanger their physical and mental health in the later stage. Therefore, it is necessary to intervene and control the dangerous behaviors of teenagers too early [12, 13].

In this study, students who had AHRB behavior at least once in three years from 2018 to 2020 were selected to intervene in the teaching of quality education sports dance class with artificial intelligence intervention in full-time ordinary primary and secondary schools and to observe the behavioral effect of the recurrence of AHRB behavior within three years after the intervention. The selected students include 9 middle schools and 24 primary schools in a city. 235 students are selected, including 112 girls and 123 boys, aged 9-15 years, with an average age of 10.6 ± 1.8 years. 65 students have one AHRB behavior, 89 students have two AHRB behaviors, and 81 students have three or more AHRB behaviors. The students are divided into groups according to their age, gender, and the number of AHRB behaviors.

When the dance class of quality education is carried out, AHRB students shall be integrated into other students in the proportion of no less than 1 : 18. For example, at least 18 normal young students shall be allocated to one intervention student selected to receive the intervention of adolescent health risk behavior in the class together, so that the selected intervention students cannot be targeted and be able to achieve “senseless intervention.”

### 3.2. Investigation Scope and Method

At present, some bad behaviors around teenagers have attracted more and more primary attention of the society, such as intentional injury; drug addiction caused by drug abuse: smoking, alcoholism, etc.; uncontrolled acts of retaliation against society; physical accidental injury caused by lack of physical exercise; and various unsafe behavior states such as personality disorder behavior with mental disorders, which directly or potentially threaten the physical and mental health of teenagers and have a certain harmful impact on the society, the parties, and their families. Various adverse phenomena endangering the health of teenagers are investigated as follows.

The article "Application of Artificial Intelligence in the Intervention of Sports on Adolescent Health Risk Behavior" was retracted in 2023. Reasons: signs of a paper mill; compromised peer review; unreliable results or conclusions.

Figure 1 shows the common bad phenomena of teenagers in the current society, such as campus violence, smoking, drinking, gambling, online games, lack of exercise, and other bad phenomena. Among them, 29.7% of the youngsters in the survey lacked the amount of exercise, and the amount of exercise of girls was significantly lower than that of boys. Secondly, the phenomenon of online games is also relatively serious, and many teenagers are trapped in it. These adverse phenomena pose a serious threat to the physical and mental health of teenagers, so it is necessary to guide teenagers to conduct behavioral intervention treatment as soon as possible.

The intervention method of adolescent health risk behavior adopts the technology of artificial intelligence sports and AHRB identification intervention. Through the in-depth study of the artificial intelligence intervention technology and analysis technology of AHRB, using the quality sports dance course combined with the sports analysis function of artificial intelligence, all AHRB behavior students carry out the same intervention measures, to observe various intervention effects of students of different ages, such as various occurrence types, recurrence types, recurrence cycle, recurrence times, and other different intervention effects of AHRB behavior of students after intervention.

## 4. Analysis of Research Results

### 4.1. Intervention Effect of Students of Different Ages

Under the artificial intelligence sports system, through the behavior intervention of the sports dance course for students of different ages: 9~10 years old, 11~12 years old, and 13~15 years old who have AHRB behavior times, we observed the recurrence of intentional injury behavior, unintentional injury behavior, mental addiction behavior, and drug addiction behavior of various types of students after intervention. The recurrence of dangerous behavior intervention in adolescents is shown in Table 1.

Table 1 shows the number of AHRB behaviors after intervention among adolescents aged 9~10, 11~12, and 13~15 years. It is found that the recurrence times of health risk behaviors of students with drug addiction and mental addiction are significantly reduced after intervention, and the recurrence times become less and less with the increase in age. The recurrence frequency of intentional injury behavior, unintentional injury behavior, and uncontrolled sexual behavior has also decreased to a certain extent. It shows that after the intervention of quality-oriented sports dance course under artificial intelligence sports, it has an obvious intervention effect on reducing the recurrence times of adolescent health risk behaviors at different ages, and the younger the age, the better the intervention effect.

The article "Application of Artificial Intelligence in the Intervention of Sports on Adolescent Health Risk Behavior" was retracted in 2023. Reasons: signs of a paper mill; compromised peer review; unreliable results or conclusions.

### 4.2. Intervention Effect of Students of Different Genders

After the intervention of sports dance course behavior of students of different genders in adolescents under artificial intelligence, observe the 3-year recurrence of adverse health hazards such as drug addiction behavior, mental addiction behavior, and intentional injury behavior. The effect of the intervention is shown in Table 2.

In order to analyze the risk behaviors of different genders in adolescents in more detail, after the intervention, visualize the recurrence times of health risk behaviors in 3 years and draw Figure 2.

Table 2 and Figure 2 show the recurrence times of dangerous behaviors of students of different genders in three years after the intervention. It is found that after the intervention of the sports dance course under artificial intelligence, the recurrence times of girls are significantly less than those of boys, and the recurrence effect of boys and girls in three years after the intervention is significantly reduced. It proves the feasibility of artificial intelligence in the intervention of sports on adolescent health risk behavior.

### 4.3. Intervention Effect of Students with Different Occurrence Times of AHRB

For the students with different AHRB occurrence times among teenagers, after the intervention of the sports dance course under artificial intelligence sports, observe the intervention effect of students with different AHRB occurrence times, as shown in Table 3.

Visualize the 3-year recurrence times after intervention with different AHRB occurrence times in adolescents, as shown in Figure 3.

Table 3 and Figure 3 show the recurrence times of adolescent students with different occurrence times of AHRB in 3 years after the intervention. It is found that the intervention effect of unintentional injury behavior, intentional injury behavior, and personality disorder behavior is obvious in the recurrence times of one time. Among the two recurrence times, the recurrence times of personality disorder behavior, uncontrolled sexual behavior, uncontrolled sexual behavior, and unintentional injury behavior also decreased significantly after intervention. Among the three recurrence times, the recurrence times of personality disorder behavior and uncontrolled sexual behavior were also the least. It is proven that the intervention can significantly reduce the recurrence times of various dangerous behaviors of adolescents, and the recurrence times are less and less, which is beneficial to the physical and mental health of adolescents.

The article "Application of Artificial Intelligence in the Intervention of Sports on Adolescent Health Risk Behavior" was retracted in 2023. Reasons: signs of a paper mill; compromised peer review; unreliable results or conclusions.

### 4.4. Occurrence of AHRB Behavior of Non-AHRB Students

In order to better analyze the application effect of artificial intelligence in the intervention of adolescent health risk behavior in sports, the students with AHRB behavior and non-AHRB students in adolescents were intervened together to observe the effect of non-AHRB students after the intervention, as shown in Table 4.

By visualizing the occurrence of AHRB behavior of non-AHRB students among teenagers, Figure 3 is obtained.

Table 4 and Figure 4 show that in the comparison between the non-AHRB students and the students who did not participate in the course intervention after the intervention, the various health risk behaviors of the non-AHRB students have been significantly reduced, and the reduction effect is obvious. It shows that non-AHRB students and students with AHRB behavior can intervene together, which will not have an adverse impact on non-AHRB students but can improve various health behaviors of non-AHRB students, which is worthy to be popularized and applied in teenagers.

## 5. Discussion on the Intervention Effect of Sports on Adolescent Health Risk Behavior

With the overall development of society and the enhancement of educational competitiveness, parents of young students have higher and higher expectations for them. In addition to the heavy study, students also have more and more pressure from their parents, society, living environment, and spirit. Excessive physical and psychological pressure not only affects their physical development but also affects the mental health of teenagers. How to promote the physical and mental health development of teenagers has become the primary concern of the current society. In order to prevent all kinds of health risk behaviors among teenagers, parents, schools, and society need to jointly find effective ways to treat teenagers' bad behaviors and intervene them as soon as possible to help teenagers form good habits of physical and mental health development, so as to reduce the adverse effects on schools, families, and society.

## 6. Discussion on the Intervention Effect of Artificial Intelligence on Adolescent Health Risk Behavior

The continuous development of artificial intelligence technology can not only bring more convenience to people's life but also realize behavior intervention in real life. For example, the intervention of teenagers' health risk behavior under artificial intelligence technology is to intervene the behavior of teenagers by using sports dance courses and artificial intelligence technology, and through the intervention of various bad behaviors of teenagers, artificial intelligence technology can reduce the risk behavior of adolescents and can predict the possible intervention results, which is conducive to the healthy development of adolescents and plays an important role in the related research of a health risk behavior intervention among adolescents in the future.

The article "Application of Artificial Intelligence in the Intervention of Sports on Adolescent Health Risk Behavior" was retracted in 2023. Reasons: signs of a paper mill; compromised peer review; unreliable results or conclusions.

## 7. Summary

Through the application of artificial intelligence in the intervention of sports on teenagers' health risk behaviors, this study uses the technical analysis of an artificial intelligence sports dance course and AHRB identification intervention to observe and compare the intervention effects of students of different ages and genders. The intervention effect of students with different ahrb occurrence times, and the effect of non ahrb students and ahrb behavior students participating in curriculum intervention. Finally, it is found that the intervention effect of sports under artificial intelligence on young students of different types, ages, and genders is obvious, which can reduce students' various unhealthy behaviors and reduce the recurrence times within 3 years. It can help non-AHRB students develop various health behaviors, significantly improve the physical and mental health of teenagers, and promote the research of artificial intelligence in the field of youth sports.

## Figures and Tables

**Figure 1:** Investigation on adverse phenomena of teenagers.

**Figure 2:** Visual chart of recurrence times of risk behavior intervention in adolescents of different genders in three years.

**Figure 3:** Visualization of the number of relapses after 3 years.

**Figure 4:** Visualization of AHRB behavior of non-AHRB students.

**Table 1:** Recurrence times of risk behavior intervention in adolescents of different ages in 3 years.

Grouping	9~10 years old	11~12 years old	13-15 years old
Unintentional injury	6.9%	4.5%	3.2%
Intentional injury	10.1%	8.4%	6.3%
Drug addictive behavior	15.4%	10.7%	6.4%
Addictive behavior	18.7%	11.4%	7.1%
Uncontrolled sexual behavior	8.6%	6.3%	2.1%
Personality disorder behavior	7.1%	5.4%	3.9‰

**Table 2:** Recurrence times of risk behavior intervention for adolescents of different genders in 3 years.

Grouping	Schoolboy	Girl student	*t*	*P*
Unintentional injury	7.5 ± 0.6	5.1 ± 0.3	7.145	0.009
Intentional injury	11.2 ± 0.4	8.4 ± 0.2	8.034	0.008
Drug addictive behavior	10.7 ± 0.5	6.9 ± 0.5	6.701	0.007
Addictive behavior	12.4 ± 0.6	9.7 ± 0.4	9.014	0.005
Uncontrolled sexual behavior	9.6 ± 0.5	8.7 ± 0.3	8.954	0.007
Personality disorder behavior	7.5 ± 0.4	5.4 ± 0.2	7.478	0.006

**Table 3:** Recurrence times of different AHRB in 3 years after intervention.

Grouping	Once	2 times	≥3 times
Unintentional injury	8.7 ± 0.5	7.1 ± 0.4	6.2 ± 0.3
Intentional injury	8.3 ± 0.4	7.6 ± 0.3	6.5 ± 0.3
Drug addictive behavior	15.3 ± 0.6	11.4 ± 0.4	8.1 ± 0.4
Addictive behavior	14.3 ± 0.5	11.7 ± 0.4	7.6 ± 0.3
Uncontrolled sexual behavior	9.3 ± 0.6	7.2 ± 0.5	5.8 ± 0.4
Personality disorder behavior	8.7 ± 0.5	6.9 ± 0.4	5.2 ± 0.3

The article "Application of Artificial Intelligence in the Intervention of Sports on Adolescent Health Risk Behavior" was retracted in 2023. Reasons: signs of a paper mill; compromised peer review; unreliable results or conclusions.

**Table 4:** AHRB behavior of non-AHRB students.

Grouping	Take a course	Did not attend the course	*t*	*P*
Unintentional injury	1.3	1.6	6.354	0.008
Intentional injury	3.2	4.6	8.147	0.007
Drug addictive behavior	2.7	3.8	6.756	0.008
Addictive behavior	12.6	15.3	9.021	0.007
Uncontrolled sexual behavior	0.8	0.9	8.247	0.008
Personality disorder behavior	5.3	6.2	7.341	0.007

## Data Availability

The data underlying the results presented in the study are available within the manuscript.
